The article "Knockdown of HSDL2 inhibits lung adenocarcinoma progression via down-regulating AKT2 expression" was published in 2020. Journal: Biosci Rep.

# Knockdown of HSDL2 inhibits lung adenocarcinoma progression via down-regulating AKT2 expression

**DOI:** 10.1042/BSR20200348

**Published:** 2020-04-07

**Authors:** Yujia Shi, Zhengdao Mao, Yanhua Huang, Yun Sun, Qi Cao, Xiaowei Yin, Jianan Huang, Qian Zhang

**Affiliations:** 1 Department of Respiratory and Critical Care Medicine, the First Affiliated Hospital of Soochow University, Suzhou 215006, Jiangsu Province, China; 2 Department of Respiratory and Critical Care Medicine, the Affiliated Changzhou No.2 People’s Hospital of Nanjing Medical University, Changzhou 213003, Jiangsu Province, China

**Keywords:** gene chip, hydroxysteroid dehydrogenase-like 2, lung adenocarcinoma, non-small cell lung cancer, prognosis

## Abstract

The aims of the present study are to investigate the role of hydroxysteroid dehydrogenase-like 2 (HSDL2) in the progression of lung adenocarcinoma and illuminate the underlying molecular mechanisms. ShRNA targeting *HSDL*2 gene (siHSDL2) was utilized to knockdown (KD) HSDL2 expression. *In vitro* and *in vivo* experiments were carried out to investigate the effect of siHSDL2 on the progression of lung adenocarcinoma. Microarray hybridization and gene expression analysis were used to investigate effect of siHSDL2 on mRNA expression profile in lung cancer cell line H1299. Our data demonstrated that HSDL2 was up-regulated in lung adenocarcinoma tissue samples (*P*<0.001). Patients with high HSDL2 expression in cancer tissues had a worse overall survival (*P*<0.001). HSDL2 KD not only inhibited the proliferation, cell cycle, apoptosis, clone-formation, invasion and migration of lung adenocarcinoma cells *in vitro* (*P*<0.05), but also suppressed the growth and metastasis *in vivo* (*P*<0.05). HSDL2 KD resulted in up-regulation of 681 genes and down-regulation of 276 genes. HSDL2 KD down-regulated the protein expression and phosphorylation of protein kinase B β (AKT2) (*P*<0.001 and *P*<0.001, respectively) and protein expression of baculoviral IAP repeat-containing 3 (BIRC3; *P=*0.001), and up-regulated the phosphorylation of ERK (*P*<0.001). Rescue experiments showed that AKT2 overexpression reversed the suppression effect of siHSDL2 on cell proliferation (*P*<0.001), invasion (*P*<0.001) and migration (*P*<0.001) significantly. HSDL2 functions as an oncogene to promote the growth and metastasis of lung adenocarcinoma via promoting the expression of AKT2.

## Background

Lung cancer has the highest mortality rate of all malignant tumors, and approximately 1.5 million people die from lung cancer every year worldwide [1]. According to the statistics of the World Health Organization, in 2025, the number of new lung cancer deaths in China will exceed 1 million each year, ranking first in the world [2]. Eighty to eighty five percent of lung cancer is non-small cell lung cancer (NSCLC), in which lung adenocarcinoma is one of the major pathological type [3]. The vast majority of patients with lung adenocarcinoma are in advanced stage at the time of initial diagnosis, and lose indications for surgery, so drug treatments become the preferred method for such patients [4]. In view of the fact that the efficacy of platinum-containing chemotherapy regimens has gradually entered a plateau and the side-effects are large, the molecular targeted drugs labeled with ‘precision treatment’ have been widely used with the advantages of high efficiency and fewer side-effects in lung adenocarcinoma [5]. Among molecular targeted drugs, epidermal growth factor receptor (EGFR) tyrosine kinase inhibitors (TKIs) are the most widely used [6]. In EGFR gene-sensitive patients with lung adenocarcinoma, the efficacy of TKIs are significantly better than conventional chemotherapy drugs [7]. However, these patients will inevitably develop TKI resistance after a period of use [8], so it is necessary to further explore tumor-driven genes and related activation signaling pathways to find new targets for molecular targeted therapy in lung adenocarcinoma.

The article "Knockdown of HSDL2 inhibits lung adenocarcinoma progression via down-regulating AKT2 expression" was published in 2020. Journal: Biosci Rep.

In the past few decades, a large number of studies have shown that abnormal lipid metabolism is a major marker of tumors [9–12]. Previous studies have shown that dehydrogenase/reductase (SDR) dysfunction plays a role in many diseases, such as Alzheimer’s disease [13,14], obesity [15], and cancer [16]. However, the functions of many SDR family members are not yet clear. Hydroxysteroid dehydrogenase-like 2 (HSDL2) is a member of the SDR family, and the HSDL2 protein consists of 418 amino acids and contains a sterol carrier protein 2 (SCP2) domain [17,18]. HSDL2 can bind to coenzyme NADPH and participates in the synthesis of cholesterol [19]. It has been found that when HSDL2 is overexpressed, intracellular cholesterol synthesis is significantly accelerated, and total cholesterol in the body is significantly increased [19]. Studies have shown that the role of HSDL2 in tumor progression is complex and influenced by the type of tumor. HSDL2 has promoting effects on tumor progression in papillary thyroid cancer [20], bladder cancer [21], ovarian cancer [22], and glioma [23], but has suppressing effects in cholangiocarcinoma [24]. At present, the role of HSDL2 in the progression of NSCLC remains unclear.

In the present study, we used short hairpin RNA (shRNA) technology to knockdown (KD) HSDL2 expression to investigate the role of HSDL2 in the progression of lung adenocarcinoma. We found that HSDL2 KD significantly suppressed the proliferation, cell cycle, clone formation, invasion and migration, and induced the apoptosis in lung adenocarcinoma cells *in vitro*. Besides, HSDL2 KD could also suppress tumor growth and metastasis in lung adenocarcinoma mouse models. Based on the results from microarray hybridization and gene expression analysis, we speculated that protein kinase B β (AKT2) is a downstream protein of HSDL2, which plays an important role in the anti-tumor process induced by HSDL2 KD. HSDL2 appears to be a novel potential target for molecular targeted therapy in lung adenocarcinoma.

The article "Knockdown of HSDL2 inhibits lung adenocarcinoma progression via down-regulating AKT2 expression" was published in 2020. Journal: Biosci Rep.

## Methods

### Patients and samples

Human lung adenocarcinoma tissues and corresponding adjacent normal tissues were obtained from 86 patients who underwent radical operations at the Department of Cardiothoracic Surgery in the Affiliated Changzhou No.2 People’s Hospital of Nanjing Medical University between January 2007 and December 2011. No patient received chemotherapy or radiotherapy prior to surgical resection. All tissues were cut off to make pathological sections and immunohistochemistry (IHC) sections. The following clinical parameters of patients were collected: gender, age, histopathology grade, lymph node invasion, TNM (tumor, lymph node, metastasis) stage and follow-up time. The detailed information of all participants were displayed in Table 1. The present study was approved by the Ethics Committee of Affiliated Changzhou No.2 People’s Hospital of Nanjing Medical University. The signed informed consents of all participants were obtained.

**Table 1:** Patients’ characteristics

Variable	Cases	HSDL2 expression		χ^2^	*P*-value
		Group low	Group high		
Gender				1.705	0.205
Male	58	13	45		
Female	28	10	18		
Age (years)				6.031	0.016
<60	41	16	25		
≥60	45	7	38		
Grade				4.662	0.047
I/II	36	14	22		
III/IV	50	9	41		
Lymph node invasion				21.931	<0.001
Non-invasion	39	20	19		
Invasion	47	3	44		
TNM stage				12.663	0.001
I/II	27	14	13		
III/IV	59	9	50		

### IHC and staining evaluation

After dewaxing and rehydration, sodium citrate (pH 6.0) was used for antigen retrieval at 120°C for 15 min. The section was then incubated in 0.3% hydrogen peroxidase for 30 min at 37°C. Subsequently, the specimens blocked with 3% BSA were incubated with anti-HSDL2 antibody (1:200, Abcam) overnight at 4°C. After incubation with anti-mouse/rabbit secondary antibody (Abcam) for 30 min at 37°C, the specimens were stained using a diaminobenzidine kit (Sigma, U.S.A.). The intensity of staining was evaluated according to the following scale: 0, no staining; 1, weak staining; 2, moderate staining; 3, strong staining [25]. The proportion of all staining tumor cells was determined and then multiplied by the staining intensity score to obtain a final semi-quantitative H score (maximum value of 300 corresponding to 100% of staining tumor cells with an overall staining intensity score of 3). The scores exhibiting less than 100 were classified as low expression and the others as high expression. All IHC images were blindly evaluated by two experienced observers, and the mean of the two determinations was used for further analysis.

The article "Knockdown of HSDL2 inhibits lung adenocarcinoma progression via down-regulating AKT2 expression" was published in 2020. Journal: Biosci Rep.

### Cell culture and transfection

Human lung cancer cell lines (H1975, A549, SK-MES-1, H1688, and H1299) and a normal human lung epithelial cell line (BEAS-2B) were obtained from the Shanghai Institutes of Biological Sciences Cell Bank (Shanghai, China). All cells were maintained in RPMI-1640 medium (Thermo Fisher Scientific) supplemented with 10% fetal bovine serum (Gibco, Thermo Fisher Scientific) and 1% penicillin/streptomycin at 37°C in a humidified incubator of 5% CO_2_. ShRNA targeting *HSDL2* gene (siHSDL2), shRNA vector, AKT2-overexpressing plasmid (plasmid AKT2), and plasmid vector were purchased from GenePharma (Shanghai, China). The sequence of shRNA targeting *HSDL2* gene was as follows: 5′-CCGGCCAGAAGCAGTTAGCAAGAAATTCAAGAGATTTCTTGCTAACTGCTTCTGGTTTTTG-3′. Luciferase vector was purchased from Promega (Wisconsin Madison, U.S.A.). All transfections were done using Lipofectamine® 2000 (Invitrogen, Thermo Fisher Scientific) according to the manufacturer’s protocols.

### Reverse transcription-quantitative polymerase chain reaction

We isolated the total RNA from cells using the TRIzol reagent (Takara Bio, Tokyo, Japan) and then reverse transcribed it into cDNA using the PrimeScript RT reagent kit (Takara Bio, Tokyo, Japan). Reverse transcription-quantitative polymerase chain reactions (RT-PCRs) were carried out using the SYBR Premix Ex Taq II (Takara Bio, Tokyo, Japan) on an ABI PRISM 7500 Sequence Detection system (Applied Biosystems, U.S.A.) according to the manufacturer’s instructions. Briefly, after an initial denaturation step at 95°C for 30 s, amplifications were conducted with 40 cycles at a melting temperature of 95°C for 5 s, and an annealing temperature of 60°C for 34 s. Human glyceraldehyde-3-phosphate dehydrogenase (GAPDH) was used as the housekeeping gene to normalize the expression level of target gene. Primers used for amplifications were as follows: 5′-AAGCCACTCAAGCAATCTATCTG-3′ (forward) and 5′-GCTCTCCATATCCGACATTCCC-3′ (reverse) for HSDL2; and 5′-TGACTTCAACAGCGACACCCA-3′ (forward) and 5′-CACCCTGTTGCTGTAGCCAAA-3′ (reverse) for GAPDH.

### Western blotting analysis

Proteins were extracted from the lysed cells using mammalian protein extraction agent (Thermo Fisher Scientific) plus halt protease inhibitor cocktail (Thermo Fisher Scientific). Protein concentrations were detected using a bicinchoninic acid assay (Thermo Fisher Scientific) according to the manufacturer’s instructions. Equal amounts of proteins were loaded on to 10% sodium dodecyl sulfate/polyacrylamide gels (SDS/PAGE) for electrophoresis. Then proteins on gels were transferred on to polyvinylidene fluoride (PVDF) membranes (Millipore, U.S.A.). After being blocked with 5% bovine serum albumin in PBST (0.1% Tween 20 in PBS) for 1 h, membranes were hybridized with primary antibodies to human HSDL2 and GAPDH at 4°C overnight. On the next day, after being washed three times with PBST for 10 min, membranes were hybridized with the corresponding secondary antibodies conjugated with horseradish peroxidase for 2 h at room temperature. Subsequently, after being washed three times with PBST for 10 min, immunoreactive proteins on the membranes were detected using ECL assay. The protein bands were visualized using SuperSignal West Pico Chemiluminescent substrate (Thermo Fisher Scientific) and quantified using ImageJ 1.50i (National Institutes of Health, Bethesda, MD, U.S.A.).

The article "Knockdown of HSDL2 inhibits lung adenocarcinoma progression via down-regulating AKT2 expression" was published in 2020. Journal: Biosci Rep.

### Cell proliferation assays

Cellomics ArrayScan VT1 Reader (Cellomics, Pittsburgh, PA, U.S.A.) was used to detect the cell proliferation. Briefly, cells in the logarithmic stage were digested and resuspended and 2,000 cells/well were seeded into 96-well plates. Since day 2, we used Cellomics ArrayScan VT1 Reader to calculate the cell number once a day at an interval of 5 days. The number of cells with green fluorescence in each scan orifice were calculated accurately. Finally, the cell proliferation curve was plotted. The 3-(4,5-dimethylthiazol-2-yl)-2,5-diphenyltetrazolium bromide (MTT) assay was also used to detect the cell proliferation. Briefly, cells in the logarithmic stage were digested and resuspended and 2000 cells/well were seeded into 96-well plates. A total of five 96-well plates were set for detecting once a day at an interval of 5 days. Since day 2, 10 μl of MTT solution (5 mg/ml) was added into each well 4 h before the termination of the culture. Following a 10-min incubation with 100 µl of dimethyl sulfoxide, the absorbance at 490 nm was measured using the Multiscan Plate Reader (Thermo Fisher Scientific). Finally, the cell proliferation curve was plotted. The experiment was repeated three times.

### Cell cycle assay

When grown to 80% confluence, cells were digested, resuspended, and centrifuged at 1200 rpm for 5 min. Then cells were washed in chilled PBS and fixed in 75% alcohol for 1 h, followed by staining with propidium iodide (50 µg/ml, Sigma–Aldrich, MO, U.S.A.) in the presence of RNase A (100 µg/ml, Fermentas, Shanghai, China). Finally, we analyzed the cell cycle using BD FACSCalibur flow cytometer (BD Biosciences, CA, U.S.A.). The experiment was repeated three times.

The article "Knockdown of HSDL2 inhibits lung adenocarcinoma progression via down-regulating AKT2 expression" was published in 2020. Journal: Biosci Rep.

### Cell apoptosis assay

An Annexin V-APC Apoptosis Detection Kit (eBioscience, CA, U.S.A.) was used to detect the cell apoptosis. Cells were digested, resuspended, centrifuged at 1500 rpm for 5 min. Then cells were washed in chilled PBS and 1× binding buffer, followed by resuspension in 1 ml of 1× staining buffer and 5 ml of Annexin V-APC into 100 ml cell suspension. The reaction was incubated in the dark for 15 min. Finally, cell apoptosis was analyzed using flow cytometry (FCM). The experiment was repeated three times.

### Colony formation assay

Cells in the logarithmic stage were digested and resuspended, and 800 cells/well were seeded into six-well plates and cultured for approximately 2 weeks. The culture medium was replaced every 3 days. Before counting, cells were fixed with 10% formaldehyde for 30 min and stained with Giemsa solution (Sigma–Aldrich, Shanghai, China) for 20 min at room temperature. Then the colony containing more than 50 cells was counted. The experiment was repeated three times.

### Transwell assay

Cell invasion was measured using cell culture inserts (24-well type, 8-μm pore size; Corning Inc., Corning, NY, U.S.A.). Cells in the logarithmic stage were digested and resuspended, and 1 × 10^5^ cells were added into the upper chambers with serum-free RPMI-1640 medium, while the lower chambers were filled with 500 µl complete RPMI 1640. After 48-h incubation, the invading cells were fixed in methanol and stained with Crystal Violet. Cells from five random fields were counted under a microscope. The experiment was repeated three times.

### Wound-healing assay

Cells in the logarithmic stage were digested and resuspended, and 50000 cells/well were seeded into six-well plates. When the cells had grown to 90% confluence, a 100-µl pipette tip was used to produce a wound at the middle of the well. The wound was photographed and measured at 0 and 24 h. The experiment was repeated three times.

### Xenograft tumor model

All the animal experiments were performed in Soochow University following the Guide for the Care and Use of Laboratory Animals (National Institutes of Health publication). The ethics approval was also obtained from Animal Ethics Committee of Soochow University. Female BALB/c-nude mice (4-week-old) were purchased from Shanghai Experimental Animal Center (Shanghai, China). In the tumor growth experiments, mice were inoculated with H1299 cells transfected with siHSDL2 or empty vector by hypodermia (4 × 10^6^/mouse). Tumor volume was calculated using the following formula: (length × width^2^) × π/6. In the tumor metastasis experiments, mice were inoculated with H1299 cells transfected with siHSDL2/empty vector and luciferase vector by tail vein (4 × 10^6^/mouse). Mice were killed by the method of cervical dislocation.

The article "Knockdown of HSDL2 inhibits lung adenocarcinoma progression via down-regulating AKT2 expression" was published in 2020. Journal: Biosci Rep.

### Imaging of luciferase activity *in vivo*

*In vivo* bioluminescence imaging was conducted to assess systemic tumor metastasis in mice utilizing an *In Vivo* Imaging System (IVIS) (PerkinElmer, Massachusetts, U.S.A.). Briefly, mice carrying luciferase vectors were injected intraperitoneally with 10 µg/g of d-Luciferin (15 mg/ml). After 10 min, the mice were anesthetized by inhalation of isoflurane (2.0 vol%). Subsequently, the mice were placed in a light-sealed chamber and the luciferase activity was imaged for 5–10 s using IVIS spectrum computed tomography (IVIS-CT) according to the manufacturer’s instructions. Photons emitted from various regions of mouse were quantified with Living Image software (PerkinElmer, Massachusetts, U.S.A.).

### Microarray hybridization and gene expression analysis

We extracted the total RNA from cells using TRIzol reagent, and test the quality with Thermo NanoDrop2000 (Thermo Fisher Scientific) and Agilent 2100 (Agilent Technologies, CA, U.S.A.). Then amplified RNA (aRNA) was prepared with qualified RNA using the GeneChip 3′ IVT Express Kit (Affymetrix, CA, U.S.A.). After purification, aRNA were fragmented and hybridized with a chip probe using a GeneChip Hybridization Wash and Stain Kit (Affymetrix, CA, U.S.A.). Subsequently, the chips were dyed. Finally, the images and raw data of the chips were scanned using the GeneChip Scanner 3000 (Affymetrix, CA, U.S.A.).

### Statistical analysis

Statistical analysis was carried out using SPSS v22.0 (SPSS Inc., Chicago, Illinois, U.S.A.). Student’s *t* test was used to analyze the difference between two groups. One-way analysis of variance (ANOVA) followed by Tukey’s test was used to compare three or more groups. Chi-square (χ^2^) test was used to analyze the correlation between the HSDL2 protein expression level and the clinical parameters of patients. The survival curves were plotted using the Kaplan–Meier method, and the difference was evaluated using the log-rank test. Each experiment was repeated three times. Data were presented as the mean ± standard deviation (SD). A *P*<0.05 was considered statistically significant.

## Results

### Expression of HSDL2 in lung adenocarcinoma tissues

IHC staining was performed on the cancer and adjacent tissues from 86 patients with lung adenocarcinoma. The cut-off value of IHC score was 100. Interobserver agreement in the assessment of IHC findings was excellent. The results showed that HSDL2 positive staining was mainly localized in the cytoplasm (Figure 1A). In 86 cancer tissues, HSDL2 was highly expressed in 63 (73.3%) tissues. In 86 adjacent tissues, HSDL2 was highly expressed in 17 (19.8%) tissues. There was a statistically significant difference in the expression of HSDL2 between cancer tissues and adjacent tissues (*P*<0.001, Figure 1B).

The article "Knockdown of HSDL2 inhibits lung adenocarcinoma progression via down-regulating AKT2 expression" was published in 2020. Journal: Biosci Rep.

**Figure 1:** Expression of HSDL2 in lung adenocarcinoma tissues and human lung cancer cell lines (**A**) IHC representative images of low and high HSDL2 expression on slides from human lung adenocarcinoma tissues and adjacent normal tissues. (**B**) Protein expression levels of HSDL2 in human lung adenocarcinoma tissues and adjacent normal tissues detected by IHC. (**C**) Kaplan–Meier survival curves for patients with lung adenocarcinoma based on HSDL2 expression in cancer tissue. (**D**) HSDL2 mRNA expression levels in human lung cancer cell lines (H1975, A549, SK-MES-1, H1688 and H1299) and normal human lung epithelial cell line (BEAS-2B). (**E**) HSDL2 mRNA expression levels in H1299 cells detected by RT-PCR. GAPDH was used as an internal control. (**F**) HSDL2 protein expression levels in H1299 cells detected by Western blot. GAPDH was used as an internal control. NC, transfected with empty vector, KD, transfected with HSDL2 shRNA vector. *P<0.05, **P<0.01, ***P<0.001. All data are presented as mean ± SD from three independent experiments.

### Relationship between HSDL2 expression and clinicopathological characteristics or prognosis in patients with lung adenocarcinoma

The expression of HSDL2 in cancer tissues was correlated with the age (χ^2^ = 6.031, *P*=0.016), grade (χ^2^ = 4.662, *P*=0.047), lymph node invasion (χ^2^ = 21.931, *P*<0.001), and TNM stage (χ^2^ = 12.663, *P*=0.001) in patients with lung adenocarcinoma, as shown in Table 1. In addition, survival analysis showed that patients with high HSDL2 expression in cancer tissues had a worse overall survival (*P*<0.001, Figure 1C). The mean survival time of patients with high HSDL2 expression was 48.6 months, while that of patients with low HSDL2 expression was 70.8 months.

### Expression of HSDL2 in lung cancer cell lines

We compared the expression levels of HSDL2 in human lung cancer cell lines (H1975, A549, SK-MES-1, H1688, and H1299) and normal human lung epithelial cell line (BEAS-2B). The results of RT-PCR using *GAPDH* as a reference gene indicated that the mRNA expression levels of HSDL2 in human lung cancer cell lines were significantly higher than that in human lung epithelial cell line (Figure 1D). The mRNA expression level of HSDL2 in H1299 cell line was highest, so H1299 cell line was selected for subsequent experiments to verify the role of HSDL2 in the progression of lung adenocarcinoma using siHSDL2. Cells in KD (KD) group was transfected with siHSDL2, and cells in negative control (NC) group were transfected with empty vector. RT-PCR and Western blotting were conducted to evaluate the transfection efficiency of siHSDL2. The results indicated that siHSDL2 can significantly inhibit the mRNA (*P*=0.007, Figure 1E) and protein (*P*=0.018, Figure 1F) expression levels of HSDL2 in H1299 cells.

The article "Knockdown of HSDL2 inhibits lung adenocarcinoma progression via down-regulating AKT2 expression" was published in 2020. Journal: Biosci Rep.

### Effect of HSDL2 KD on proliferation, cell cycle, and apoptosis of H1299 cells

We used the Cellomics ArrayScan VT1 Reader and MTT assay to detect the proliferation of H1299 cells in two groups for five consecutive days. The results showed that the proliferation rate of H1299 cells in the KD group was significantly inhibited compared with that in NC group (on 5th day, *P*<0.001, Figure 2A,B). The cell cycle of H1299 cells in two groups was detected by FCM. As showed in Figure 2C, after transfection of siHSDL2, the portion of H1299 cells in the S phase was significantly increased (*P*=0.001), however, the portion in the G_2_/M phase was significantly decreased (*P*=0.016). The apoptosis of H1299 cells in two groups was also detected by FCM. After transfected with siHSDL2, the apoptosis rate of H1299 cells was significantly increased (*P*=0.003, Figure 2D).

**Figure 2:** Effect of HSDL2 KD on proliferation, cell cycle, and apoptosis of H1299 cells (**A**) Cellomics ArrayScan VT1 Reader was used to detect the effect of siHSDL2 on the proliferation of H1299 cells. (**B**) MTT assay was also performed to analyze the effect of siHSDL2 on the proliferation of H1299 cells. (**C**) FCM was used to detect the effect of siHSDL2 on the cell cycle of H1299 cells. (**D**) FCM was used to detect the effect of siHSDL2 on the apoptosis of H1299 cells. NC, transfected with empty vector; KD, transfected with HSDL2 shRNA vector. *P<0.05, **P<0.01, ***P<0.001. All data are presented as mean ± SD from three independent experiments.

### Effect of HSDL2 KD on clone-formation, invasion, and migration of H1299 cells

The result from colony formation assay showed that the H1299 cells transfected with siHSDL2 has fewer colonies (*P*=0.007, Figure 3A). Cell invasion and migration was measured using transwell assay and wound-healing assay, respectively. By comparing the KD group with the NC group, it was demonstrated that siHSDL2 transfection significantly inhibited the H1299 cell invasion and migration (*P*<0.001, Figure 3B,C).

**Figure 3:** Effect of HSDL2 KD on clone-formation, invasion, and migration of H1299 cells (**A**) Colony formation assay was used to detect the effects of siHSDL2 on the clone-formation of H1299 cells. (**B**) Transwell assay was utilized to detect the effects of siHSDL2 on the invasion of H1299 cells. Magnification ×200. (**C**) Wound-healing assay was utilized to detect the effects of siHSDL2 on the migration of H1299 cells. NC, transfected with empty vector; KD, transfected with HSDL2 shRNA vector. **P<0.01, ***P<0.001. All data are presented as mean ± SD from three independent experiments.

The article "Knockdown of HSDL2 inhibits lung adenocarcinoma progression via down-regulating AKT2 expression" was published in 2020. Journal: Biosci Rep.

### Effect of HSDL2 KD on the growth of tumor

Mouse tumor models were established by endermic injection of H1299 cells. Twelve female mice (4-week-old) were randomly and equally divided into two groups: NC and KD groups. The mice in NC group were injected with H1299 cells transfected with empty vector and the mice in KD group were injected with H1299 cells transfected with siHSDL2. The length and width of the tumor were first measured on the 22nd day after inoculation, and then measured every other day for a total of five times. The growth curves of the two groups were plotted and compared. The results showed that the tumor volume proliferation of the KD group was slower than that of the NC group (on 9th day, *P*=0.006, Figure 4A). After the last measurement of the volume, the mice were immediately killed and the tumor mass was weighed. Comparing the tumor weight of the two groups, we found that the tumor weight in KD group was lighter than that in NC group (*P*=0.006, Figure 4B).

**Figure 4:** Effect of HSDL2 KD on the growth of tumor models Mouse tumor models were established by endermic injection of H1299 cells transfected with empty vector (NC) or HSDL2 shRNA vector (KD). (**A**) Tumor volume of the two groups of mice was first measured on the 22nd day after inoculation, and then measured every other day for a total of five times. (**B**) After the last measurement of the volume, the two groups of mice were immediately killed and the tumor mass was weighed. **P<0.01. All data are presented as mean ± SD from six mice.

### Effect of HSDL2 KD on the metastasis of tumor

Mouse tumor models used in this experiment were generated by tail intravenous injection of H1299 cells. Twenty female mice (4-week-old) were randomly and equally divided into two groups: NC and KD groups. The mice in NC group were tail intravenous injected with H1299 cells transfected with empty vector and luciferase vector, and the mice in KD group were tail intravenous injected with H1299 cells transfected with siHSDL2 and luciferase vector. Then the mice were weighed weekly. The results showed that there was no statistical difference in body weight between the groups (Figure 5A). In the 7th week, the body luciferase activity of the mice was detected. The results showed that the body luciferase activity of the KD group was decreased compared with the NC group (*P*=0.005, Figure 5B). Two groups of mice were dissected in the 7th week to assess their lung and liver metastasis. In the NC group, ten mice had lung metastasis, the metastasis rate was 100%, and each had a large number of metastases. In the KD group, two mice had lung metastasis, the metastasis rate was 20%, and only a small number of metastases were present. Since the lungs of the NC group were full of metastases, counting statistics could not be performed. In view of this, we indirectly assess the severity of lung metastases by weighing the lungs. The results showed that when compared with the NC group, the lung weight of the KD group was lighter (*P*<0.001, Figure 5C), suggesting that the KD group had more lung metastases. Surprisingly, in the NC and KD groups, none of the mice had liver metastasis.

The article "Knockdown of HSDL2 inhibits lung adenocarcinoma progression via down-regulating AKT2 expression" was published in 2020. Journal: Biosci Rep.

**Figure 5:** Effect of HSDL2 KD on the metastasis of tumor models Mouse tumor models were generated by tail intravenous injection of H1299 cells transfected with empty vector (NC) or HSDL2 shRNA vector (KD). (**A**) Photo of mice in the 7th week. Two groups of mice were weighed and compared weekly. (**B**) Body luciferase activity of the two groups of mice were detected and compared in the 7th week. (**C**) Lungs from the two groups of mice dissected in the 7th week were weighed and compared. ns, no significance; **P<0.01, ***P<0.001. All data are presented as mean ± SD from ten mice.

### Effect of HSDL2 KD on mRNA expression profile in H1299 cells

To further reveal the molecular mechanism of HSDL2 in the progression of lung adenocarcinoma, we looked for the downstream signaling pathways regulated by HSDL2 using gene chips (three replicate chips). Bioinformatics analysis based on gene chips showed that 681 genes were up-regulated while 276 genes were down-regulated in KD group compared with NC group (Figure 6A). The differential genes were subjected to enrichment analysis based on the genetic information of all pathways in KEGG and BIOCARTA. After sorting according to the *P*-value, the top ten gene sets were shown in Figure 6B. We screened several potential downstream target genes of HSDL2 from the cancer-related set and cell apoptosis-related set, and then verified them using Western blotting analysis. The results showed that compared with NC group, AKT2 protein expression and its phosphorylation (p-AKT2) were both significantly down-regulated (*P*<0.001 and *P*<0.001 respectively, Figure 6C), baculoviral IAP repeat-containing 3 (BIRC3) protein expression was also down-regulated (*P*=0.001, Figure 6C), and phosphorylation of extracellular signal-related kinase (p-ERK) was up-regulated (*P*<0.001, Figure 6C) in KD group. We additionally selected another cell line H1688 that highly expresses HSDL2 for knockout experiments, and examined the AKT2 protein expression and its phosphorylation using Western blot to verify whether HSDL2 and AKT2/p-AKT2 is correlated in different cell lines. The results showed that AKT2 protein expression and its phosphorylation can also be down-regulated by siHSDL2 in H1688 cells (*P*<0.001 and *P*<0.001, respectively, Figure 6D).

The article "Knockdown of HSDL2 inhibits lung adenocarcinoma progression via down-regulating AKT2 expression" was published in 2020. Journal: Biosci Rep.

**Figure 6:** Effect of HSDL2 KD on mRNA expression profile and downstream proteins expression in H1299 cells (**A**) The graph of KD group and NC group which were clustered by using the expression profile of differential genes screened with fold change > 1.5 and FDR < 0.05 as standard. In the cluster analysis graph, each column represented a sample (X2642.1-3 represented the three replicate groups of NC, X2643.1-3 represented the three replicate groups of KD), each row represented a differential gene; the upper tree structure was based on the expression profile of the differential genes, aggregation or classification of all samples; the left tree structure represented the difference of genes. Red color indicates the relative increase in gene expression, green color indicates that gene expression is relatively down-regulated, black color indicates no significant change of gene expression, and gray color indicates that the signal intensity of the gene is not detected. (**B**) The significant enrichment of the differentially expressed genes in disease and function. The abscissa is the path name, and the ordinate is the level of significance of enrichment (base 10 negative logarithmic transformation). (**C**) The effects of siHSDL2 on the protein expression levels of potential downstream genes of HSDL2 in H1299 cells detected by Western blot. (**D**) The effects of siHSDL2 on AKT2 protein expression and its phosphorylation in H1688 cells detected by Western blot. GAPDH was used as an internal control in the Western blot analysis. NC: transfected with empty vector, KD: transfected with HSDL2 shRNA vector. ns, no significance; **P<0.01, ***P<0.001. Data are presented as mean ± SD from three independent experiments.

### The value of AKT2 for the function of HSDL2

We hypothesized that the suppression effect of siHSDL2 on the progression of lung adenocarcinoma depends on the AKT2 expression level. To verify this hypothesis, we conducted some rescue experiments. First, we transfected siHSDL2 vector and AKT2 plasmid vector into H1299 cells. Then, the cell proliferation, invasion, and migration were detected using MTT, transwell, and wound-healing assay. By comparing the siHSDL2 group with the control group, we found that the siHSDL2 significantly inhibited cell proliferation (on 5th day, *P*<0.001, Figure 7A), invasion (*P*<0.001, Figure 7B), and migration (*P*<0.01, Figure 7C), which were consistent with previous experiments. By comparing the AKT2 group with the control group, the AKT2 plasmid significantly promoted cell proliferation (on 5th day, *P*=0.002, Figure 7A), invasion (*P*<0.001, Figure 7B), and migration (*P*<0.05, Figure 7C). By comparing the siHSDL2+AKT2 group with the siHSDL2 group, rescue experiments showed that AKT2 plasmid significantly reversed the suppression effects of siHSDL2 on cell proliferation (on fifth day, *P*<0.001, Figure 7A), invasion (*P*<0.001, Figure 7B), and migration (*P*<0.001, Figure 7C).

The article "Knockdown of HSDL2 inhibits lung adenocarcinoma progression via down-regulating AKT2 expression" was published in 2020. Journal: Biosci Rep.

**Figure 7:** Rescue experiments investigating the value of AKT2 for the functions of HSDL2 (**A**) MTT assay was performed to analyze the effects of siHSDL2 and/or plasmid AKT2 on the proliferation of H1299 cells. (**B**) Transwell assay was utilized to analyze the effects of siHSDL2 and/or plasmid AKT2 on the invasion of H1299 cells. Magnification ×200. (**C**) Wound-healing assay was performed to detect the effects of siHSDL2 and/or plasmid AKT2 on the migration of H1299 cells. *P<0.05, **P<0.01, ***P<0.001, vs control group; ^###^*P*<0.001, vs siHSDL2 group. All data are presented as mean ± SD from three independent experiments.

## Discussion

In the present study, results from IHC indicated that high HSDL2 expression is a poor prognosis factor in patients with lung adenocarcinoma. The cell cycle assay showed that siHSDL2 could block the progression of H1299 cells from S phase to G_2_/M phase and arrest the cell cycle in S phase, which caused mitotic arrest and apoptosis. This result is consistent with that from the study by Zeng et al. [20], and also agrees with the results from our proliferation assay and apoptosis assay which showed that siHSDL2 inhibited the proliferation and promoted apoptosis of H1299 cells. Results from *in vitro* experiments disclosed that HSDL2 KD inhibited the growth and metastasis of lung adenocarcinoma. Several previous studies investigating the effects of HSDL2 in other malignant tumors have also confirmed the anti-tumor effects of HSDL2 KD [20–23]. But unfortunately, the molecular mechanism underlying the role of HSDL2 on tumor progression has not been further explored in these studies.

In our study, we not only examined the biological functions of HSDL2, but also preliminarily explored the specific molecular mechanism that regulated these functions. By detecting the protein levels of genes with significant expression differences provided by bioinformatics analysis based on gene chips, we found that HSDL2 KD down-regulated the expression of AKT2 and BIRC3, inhibited the activation of AKT2, and promoted the activation of ERK. Because the AKT2 protein expression and its phosphorylation were both significantly suppressed by siHSDL2, we further conducted rescue experiments to verify the value of AKT2 for the function of HSDL2, which showed that the suppression effect of siHSDL2 on the progression of lung adenocarcinoma cells depended on the AKT2 expression level. It indicated that AKT2 is a key molecule in the downstream signaling pathway of HSDL2.

The article "Knockdown of HSDL2 inhibits lung adenocarcinoma progression via down-regulating AKT2 expression" was published in 2020. Journal: Biosci Rep.

A previous study performed by Zeng et al. [20] investigated the role of HSDL2 in papillary thyroid cancer using similar research methods to ours. They conducted *in vitro* experiments to confirm that HSDL2 KD suppressed the proliferation and cycle, and promoted the apoptosis of papillary thyroid cancer cells. Their results from *in vivo* experiments showed that HSDL2 KD significantly suppressed the tumor growth. These results are highly consistent with ours. However, their bioinformatics analysis based on gene chips showed that AKT3, nuclear factor of activated T-cells, cytoplasmic 2 (NFATc2), and protein phosphatase 3 catalytic A (PPP3CA) were potential targets of HSDL2 in papillary thyroid cancer. Our results showed that AKT2, BIRC3, and ERK are potential targets of HSDL2 in lung adenocarcinoma. We hypothesized that HSDL2 has different targets in different tumors, or that these genes are all targets of HSDL2 and are involved in regulating tumor progression together. Unfortunately, they did not further investigate the value of AKT3, NFATc2, or PPP3CA for the function of HSDL2, but we conducted rescue experiments confirming that AKT2 plasmid significantly reversed the suppression effects of siHSDL2 on lung adenocarcinoma cell proliferation, invasion, and migration. In addition, we further detected the effects of HSDL2 KD on lung and liver metastasis of lung adenocarcinoma. Therefore, our research is relatively comprehensive.

AKT2 is an important subtype of protein kinase B (AKT) and is an important factor in the phosphoinositide 3-kinase (PI3K)/AKT signaling pathway. AKT2 regulates the signal transduction initiated by PI3K, which is involved in many cellular processes including cell cycle regulation, apoptosis initiation, tumor angiogenesis, lymphangiogenesis, and cell invasion [26–28]. Transfection of human AKT2 cDNA into human breast and ovarian cancer cells increased the invasion and metastasis ability of tumor cells by up-regulating integrin β12 [29]. BIRC3 is one of the inhibitors of apoptosis proteins (IAPs) and can block cell apoptosis by directly inhibiting the activities of downstream caspase-3 and caspase-7 or by inhibiting the activities of caspase-9 and its precursor [30,31]. ERK belongs to mitogen-activated protein kinases (MAPKs) which play an important role in many cellular processes including cell proliferation, differentiation, and apoptosis [32]. The activation of ERK is involved in growth arrest and apoptosis via reactive oxygen species (ROS) generation [33,34]. Previous studies have shown that the phosphorylation level of ERK is inversely related to AKT2 and BIRC3 expression [35–37]. However, it is still unclear whether ERK is located downstream of AKT2 or BIRC3. Based on the experimental results mentioned above, we hypothesized that HSDL2 can promote the expression of AKT2 which up-regulates the expression of BIRC3, and then inhibits the phosphorylation of ERK. Of course, more further experiments are needed to verify this hypothesis.

The article "Knockdown of HSDL2 inhibits lung adenocarcinoma progression via down-regulating AKT2 expression" was published in 2020. Journal: Biosci Rep.

There were still several limitations in the present study. First, only one cell line was used for the experiments. Lung adenocarcinoma cell line contains multiple types, and H1299 cell is only one of the types. Therefore, one cell line may be not sufficient to represent all lung adenocarcinoma cell lines. And two or more cell lines are necessary for mutual verification of experimental results. Second, AKT2, BIRC3, and ERK are downstream molecules of HSDL2, but the regulatory relationship of the three molecules remains to be explored. We only theorized the relationship between the three, and it is necessary to conduct blocking experiments to verify this theory. Third, rescue experiments contain only *in vitro* experiments of proliferation, invasion, and migration, and may be slightly insufficient for validation of AKT2 value. Finally, we only knocked down HSDL2 expression using shRNA targeting *HSDL2* gene. The possibility about potential off-target effect from shRNA might exist. A rescue experiment through transfecting shRNA resistant HSDL2 plasmid should have been performed to prove no off-target effect from shRNA.

## Conclusions

The present study is the first research investigating the role of HSDL2 in lung adenocarcinoma. *In vitro* and *in vitro* experiments showed that HSDL2 KD inhibited the growth and metastasis of lung adenocarcinoma. AKT2 is a key molecule in the downstream signaling pathway of HSDL2. HSDL2 is a novel potential target for molecular targeted therapy in lung adenocarcinoma.

## Data Availability

The datasets used and/or analyzed during the current study are available from the corresponding author on reasonable request.

## Abbreviations

AKT: protein kinase B
AKT2: protein kinase B β
aRNA: amplified RNA
BIRC3: baculoviral IAP repeat-containing 3
EGFR: epidermal growth factor receptor
FCM: flow cytometry
GAPDH: glyceraldehyde-3-phosphate dehydrogenase
HSDL2: hydroxysteroid dehydrogenase-like 2
IHC: immunohistochemistry
IVIS: *In Vivo* Imaging System
KD: knockdown
MTT: 3-(4,5-dimethylthiazol-2-yl)-2,5-diphenyltetrazolium bromide
NC: negative control
NFATc2: nuclear factor of activated T-cells, cytoplasmic 2
NSCLC: non-small cell lung cancer
PI3K: phosphoinositide 3-kinase
PPP3CA: protein phosphatase 3 catalytic A
RT-PCR: reverse transcription-quantitative polymerase chain reaction
TKI: tyrosine kinase inhibitor
TNM: tumor, lymph node, metastasis
